The article "Overexpression of long non-coding RNA LINC00982 suppresses cell proliferation and tumor growth of papillary thyroid carcinoma through PI3K-ATK signaling pathway" was published in 2019. Journal: Biosci Rep.

# Overexpression of long non-coding RNA LINC00982 suppresses cell proliferation and tumor growth of papillary thyroid carcinoma through PI3K-ATK signaling pathway

**DOI:** 10.1042/BSR20191210

**Published:** 2019-07-12

**Authors:** Debin Xu, Jichun Yu, Shimin Zhuang, Shuyong Zhang, Zhengdong Hong, Chunlei Yuan

**Affiliations:** 1 Department of Thyroid and Neck Surgery, the Second Affiliated Hospital of Nan Chang University, 1 MinDe Road, Nanchang, Jiangxi 360006, People’s Republic of China; 2 Departments of Otolaryngology-Head & Neck Surgery, The Sixth Affiliated Hospital of Sun Yat-sen University, 26YuanChun Two Road, Guangzhou, Guangdong 510655, People’s Republic of China; 3 Department of Urinary Surgery, the Second Affiliated Hospital of Nan Chang University, 1 MinDe Road, Nanchang, Jiangxi 360006, People’s Republic of China; 4 Department of Breast Surgery, the Second Affiliated Hospital of Nan Chang University, 1 MinDe Road, Nanchang, Jiangxi 360006, People’s Republic of China

**Keywords:** apoptosis, cell proliferation, LINC00982, papillary thyroid carcinoma, PI3K/AKT

## Abstract

Long non-coding RNAs (lncRNAs) have been widely reported that involved in human cancers, including papillary thyroid carcinoma (PTC). The present study aims to investigate the biological role of LINC00982 in PTC. The mRNA expression of LINC00982 in human PTC tissues was detected using qPCR. Moreover, Kaplan–Meier method was performed to analyze the internal relevance between LINC00982 expression and overall survival (OS) rate of patients with PTC. In addition, gain- and loss-of-functions assays were performed to detect the effects of LINC00982 on the cell proliferation and migration in PTC cells. Furthermore, western blot assay was used to measure the alteration expression levels of apoptosis relative proteins and the relative protein involved phosphatidylinositol 3-kinase (PI3K)/AKT signaling pathway. Finally, a xenograft model was used to analyze the antitumor role of LINC00982 *in vivo*. Here, we found that LINC00982 was decreased in human PTC tissues. Patients with decreased LINC00982 expression levels had a reduced OS (*P*=0.0019) compared with those with high LINC00982 expression levels. Overexpression of LINC00982 suppressed the proliferation and migration of BHT101 and B-CPAP cells and promoted cell apoptosis. Knockdown of LINC00982 promoted the proliferation and migration of BHT101 and B-CPAP cells and induced cell apoptosis. Moreover, *in vivo* assay showed that overexpression of LINC00982 could suppress the growth of PTC. Finally, LINC00982 could regulate the activity of PI3K/AKT signaling pathway *in vitro* and *in vivo*. Taken together, our findings demonstrated that overexpression of LINC00982 could suppress cell proliferation and induce cell apoptosis by regulating PI3K/AKT signaling pathway in PTC.

The article "Overexpression of long non-coding RNA LINC00982 suppresses cell proliferation and tumor growth of papillary thyroid carcinoma through PI3K-ATK signaling pathway" was published in 2019. Journal: Biosci Rep.

## Introduction

During the past decades, the morbidity and mortality of thyroid cancer are continuously increasing [1]. Thyroid cancer has gradually become a prevalent malignancy in endocrine system [2]. According to the follicular origin, thyroid cancer is divided into four subtypes, including follicular thyroid cancer, papillary thyroid cancer (PTC), partially differentiated thyroid cancer or anaplastic thyroid cancer [3]. The PTCs account approximately for 80% of all thyroid tissue malignancies and mainly occur in children and young women [4]. Because of the different pathological patterns of thyroid cancers with each cancer, the 5-year survival rate of PTC patients is less than 60% [5]. Therefore, investigating the underlying mechanism of occurrence and development of thyroid cancer may provide potential effective therapeutic strategies.

Long non-coding RNAs (lncRNAs) are a group of RNAs with a length of more than 200 nts. During the past decades, the role of lncRNAs in carcinogenesis has been widely reported, and lncRNAs have been regarded as crucial regulators involved in human cancers playing as tumor suppressors or oncogenes [6, 7]. LncRNAs are often dysregulated in human cancers and could promote tumor growth, migration and/or invasion and induce cell apoptosis, including hepatocellular carcinoma [8], non-small cell lung cancer [9], cervical cancer [10], renal cell carcinoma [11], pancreatic cancer [12], as well as PTC [13, 14]. The long intergenic non-protein coding RNA 982 (LINC00982) was found dyregulated in different human cancers. In gastric cancer, Kaplan–Meier survival analysis showed that LINC00982 was an independent prognostic factor for gastric cancer patients’ overall survival (OS) and overexpression of LINC00982 could inhibit gastric cancer growth [15]. Also, Fei et al. found that LINC00982 was decreased in human gastric cancer and decreased LINC00982 expression was negatively correlated with advanced TNM stage, invasion depth, and regional lymph node metastasis [16]. Lv et al. found that low expression level of LINC00982 was associated with poor survival in lung adenocarcinoma [17]. In renal cancer, overexpression of LINC00982 could inhibit cell proliferation and induce apoptosis of renal cancer cells, and also could regulate the phosphatidylinositol 3-kinase (PI3K)/AKT signaling pathway [18]. Although LINC00982 was found might play as a tumor suppressor in human cancers, the underlying mechanisms of LINC00982 in occurrence and development of PTC are not reported.

In our present study, we aim to analyze the clinical significance and functions of LINC00982 in PTC. Herein, we demonstrated that down-expression of LINC00982 was a characteristic molecular change in PTC and analyzed the potential relationship between LINC00982 expression level in tumor tissues and clinicopathological features of PTC. Additional, we also investigated the effects of altered LINC00982 on the phenotypes of PTC cells *in vitro* and *in vivo*. Our data suggest that LINC00982 may represent a novel indicator of poor prognosis in PTC and may play as a potential therapeutic target for diagnosis and therapy.

The article "Overexpression of long non-coding RNA LINC00982 suppresses cell proliferation and tumor growth of papillary thyroid carcinoma through PI3K-ATK signaling pathway" was published in 2019. Journal: Biosci Rep.

## Materials and methods

### Tissue samples and cell lines

Total 68 PTC tissues and corresponding pericarcinomatous tissues were obtained from the Second Affiliated Hospital of Nan Chang University. The patients, who collected for this study, were identified as PTC through pathological examination according to the International Federation of Obstetrics and Gynecology (FIGO) criteria and did not receive any chemotherapy or radiotherapy before the surgery. Clinical pathology information for all patients is shown in Table 1. Written informed consents were received from all participators and this study was approval by the Ethics Committee of the Second Affiliated Hospital of Nan Chang University in accordance with the Declaration of Helsinki. All the samples were snap-frozen and maintained at −80°C.

**Table 1:** Clinicopathological characteristics and LINC00982 expression in 68 patient samples of PTC

Clinical parameter	Number of cases (%)
**Age (years)**	
<50	40 (58.82)
>50	28 (41.18)
**Gender**	
Male	40 (58.82
Female	28 (41.18)
**T stage**	
T1-T2	37 (54.41)
T3-T4	31 (45.59)
**LNM**	
Yes	35 (51.47)
No	33 (48.53)
**TNM**	
I/II	31 (45.59)
III/IV	37 (54.41)
**Multifocality**	
Yes	33 (48.53)
No	35 (51.47)

Abbreviation: LNM, lymph node melanomametastasis.

PTC cell lines BHT101 and B-CPAP were purchased from American Type Culture Collection (Rockville, MD, U.S.A). Cell lines were cultured in Dulbecco’s Modified Eagle’s Medium (DMEM) (GIBCO-BRL) medium containing 10% FBS (Gibco, CA, U.S.A) and 1% penicillin–streptomycin (100 U/ml penicillin and 100 mg/ml streptomycin) in a humidified atmosphere at 37°C with 5% CO_2_.

### Cell transfection

The LINC00982 overexpression plasmids pcDNA4.0-LINC00982 and control plasmids pcDNA 4.0 were obtained from a commercial manufacturer (Vipotion, Guangzhou), the LINC00982 interfering plasmids siLINC00982 (Target sequence 5′-CCAGGCACAGGUAACUCTT-3′) and control interfering plasmids siCTRL (Traget sequence 5′-UUCUCCGAACGUGUCACGUTT-3′) were obtained from GenePharma (Shanghai, China). About 1 × 10^5^ cells were seeded in 24-well plates and incubated for 24 h, then cells were transfected with 2 μg plasmids using Lipofectamine 3000 (Invitrogen, Carlsbad, CA, U.S.A.) in serum-free medium in accordance with the manufacturer’s instructions. The transfection efficiency is more than 85%. The transfected cells were cultured with medium contained 1 μg/ml puromycin for 48 hs, and then cultured in the medium contained 5 μg/ml puromycin to construct stable cell lines using for *in vivo* experiments.

The article "Overexpression of long non-coding RNA LINC00982 suppresses cell proliferation and tumor growth of papillary thyroid carcinoma through PI3K-ATK signaling pathway" was published in 2019. Journal: Biosci Rep.

### RNA extraction and quantitative real-time PCR analysis

Total RNAs from tissue samples or cultured cells were extracted using TRIzol reagent (Invitrogen Inc., U.S.A.) and quantitated using a NanoDrop2000 (Thermo Scientific, U.S.A.). Total of 2 μg RNA was used for reverse transcription reaction and cDNA synthesis using M-MLV Reverse Transcriptase (Promega, U.S.A.). SYBR Green Real-time Master Mix (TOYOBO, Japan) was used for quantitative real-time PCR (qRT-PCR) analyses. The conditions of thermal cycling were illustrated as follows: 94°C for 2 min followed by 40 cycles at 94°C for 20 s, and at 58°C for 20 s. All primers were synthesized from Sangon Biotech (Shanghai, China). GAPDH was taken as the internal control. The LINC00982 primers were 5′-AAGTCGTGCTGAGTGTCTGG-3′ (forward) and 5′-CACAACGTGCCACGAACAAT-3′ (reverse). The GAPDH primers were 5′-TGTTCGTCATGGGTGTGAA-3′ (forward) and 5′-ATGGCATGGACTGTGGTCAT-3′ (reverse). Applied Biosystems 7500 Sequence Detection system (ABI, U.S.A.) was used for qRT-PCR and data collection. 2^−ΔΔ*C*^T method was used to analyze the relative fold changes.

### Western blot analysis

Western blot analysis was performed as previously reported [19]. Briefly, total proteins were exacted using RIPA buffer (Beyotime Biotechnology, Shanghai, China) and protein concentrations were quantitated using BCA Kit (Solarbio, Beijing). Total 20 μg total proteins were segregated by 10% SDS/PAGE (Genscript, Nanjing, China) and transferred onto a PVDF membrane (Millipore, MA, U.S.A.). Subsequently, the membrane was incubated with anti-PI3K (1:2000, ab140307), anti-AKT (1:10000, ab179463), anti-AKT (phospho T308, 1:800, ab38449), anti-Bax (1:5000, ab32503), anti-Bcl-2 (1:2000, ab182858), anti-Cyclin D1 (1:5000, ab40754), anti-p21 (1:8000, ab109520), and anti-GAPDH (1:10000, ab181602) at 4°C overnight and with Goat Anti-Mouse IgG H&L (HRP, 1:2000, ab6789) or Goat Anti-Rabbit IgG H&L (HRP, 1:2000, ab6721) at 37°C for 1 h. Next, ECL (Millipore, MA, U.S.A.) was applied for chemiluminescence detection. The immunoblot signal was quantitated with ImageJ software.

### CCK-8 assay

About 1 × 10^4^ transfected PTC cells were seeded in 96-well plates. Cell viability was evaluated with Cell Counting Kit-8 (CCK-8, Dojindo, Japan) at different time points (24, 48, and 72 h) after seeding. After treated with CCK-8 at 37°C for 1 h, PTC cells were used to measure the absorbency at 450 nm using Universal Microplate Spectrophotometer (Bio-Tek Instruments, Inc., Winooski, VT, U.S.A.).

The article "Overexpression of long non-coding RNA LINC00982 suppresses cell proliferation and tumor growth of papillary thyroid carcinoma through PI3K-ATK signaling pathway" was published in 2019. Journal: Biosci Rep.

### EdU incorporation assay

EdU cell proliferation kit (Ribo, Guangzhou, China) was used to analyze the proliferation ability of transfected BHT101 and B-CPAP cells in accordance with the manufacturer’s instructions. In briefly, 2 days after transfection, cells were treated with EdU for 2 h, then cells were fixed with 4% formaldehyde, and stained as previously reported [20]. The ratio of EdU-positive cells was calculated as EdU-stained cells/DAPI-stained cells. All experiments were performed in triplicate.

### Colony formation assay

The transfected BHT101 and B-CPAP cells were digested and placed into a six-well plate at a concentration of 500 cells/well, and cells were incubated for 14 days in DMEM medium containing 10% FBS. To visualize and count the colonies, methanol and 0.5% crystal violet (Sigma) were separately used to fix and stain colonies. At the end of each experiment, the cells were fixed with 4% paraformaldehyde and stained with 0.5% crystal violet (Sigma, U.S.A.). Cell colonies were visualized and counted under an inverted microscope. The experiment was performed in triplicate.

### Flow cytometry

Cell cycle distribution and cell apoptosis were determined using cell cycle staining kit (MultiSciences, Shanghai, China) and Annexin-V FITC/PI apoptosis detection kit (Life Technologies, Waltham, MA, U.S.A.) in accordance with the manufacturer’s instruction, respectively. For cell cycle distribution, the transfected BHT101 and B-CPAP cells were stained with PI solution for 30 min and then analyzed by flow cytometry on a FACScan (BD, Biosciences, U.K.). For cell apoptosis detection, the transfected BHT101 and B-CPAP cells were harvested and stained with Annexin-V FITC/PI apoptosis detection kit and then analyzed using a FACScan (BD, Biosciences, U.K.). Annexin-V(+)/PI(−) represented the cells in early apoptosis and Annexin-V(+)/PI(+) represented the cells in late apoptosis.

### Cell migration and invasion assay

The cell migration and invasion assays were performed using the 24-well transwell chambers in accordance with the manufacturer’s protocol, and were performed as previously reported [21]. The experiment was performed in triplicate.

### Xenograft tumor model

A total of 30 8-week-old BALB/c nude mice with an average weight of 20 g were obtained from Beijing Vital River Laboratory Animal Technology Co., Ltd (Beijing, China), and were fed in standard conditions. Flank tumors were established by injecting 5 × 10^6^ transfected BHT101 cells in 100 μl of PBS into the subcutaneous flanks of nude mice. Tumor dimensions were measured at each time point using the electronic calipers. Tumor volumes were calculated by the following formula: L × W × W × 0.5, L: the largest diameter, W: the perpendicular diameter. About 28 days after implantation, the mice were euthanized using 20% CO_2_ exposure for 10 min. The tumors were resected for further analysis. The animal protocol was maintained in accordance with the guidelines of the animal care committee of the Second Affiliated Hospital of Nan Chang University, and all procedures were approved by the ethics committee of the Second Affiliated Hospital of Nan Chang University.

The article "Overexpression of long non-coding RNA LINC00982 suppresses cell proliferation and tumor growth of papillary thyroid carcinoma through PI3K-ATK signaling pathway" was published in 2019. Journal: Biosci Rep.

### Statistical analysis

All experiments were performed at least three independent times. Data are processed using SPSS 20.0 statistical software (SPSS Inc, U.S.A.) and presented as the mean ± S.D. A paired or unpaired student’s *t*-test or one-way ANOVA was used for statistical comparison between means where applicable. Survival curve was generated with Kaplan–Meier method. The p-values <0.05 were considered statistically significant.

## Results

### The expression of LINC00982 and its correlation with the clinical parameters in patients with PTC

The expression levels of LINC00982 in PTC tissues and adjacent pericarcinomatous tissues were detected using qRT-PCR. As shown in Figure 1A, the expression of LINC00982 was found significantly decreased in PTC tissues compared with corresponding non-tumor tissues (*P<*0.001). Furthermore, the correlation between LINC00982 expression level and the clinical features of PTC patients was analyzed. It was revealed that lower expression of LINC00982 was closely related with high T stage (*P<*0.01, Figure 1B), advanced TNM stage (*P<*0.001, Figure 1C), positive lymph node metastasis (*P<*0.01, Figure 1D), and with multifocality (*P<*0.01, Figure 1E). However, LINC00982 expression level was not associated with other parameters, such as age and gender (data not shown). Moreover, Kaplan–Meier method was carried out to verify the prognostic value of LINC00982 for PTC patients. High expression of LINC00982 was positively correlated with the OS rate of PTC patients (*P=*0.0019, Figure 1F). Our results indicated the potential of LINC00982 expression as a novel biomarker for PTC and might help with diagnosis and monitor therapeutic efficacy.

**Figure 1:** The expression of LINC00982 and its correlation with the clinical parameters in patients with PTC (**A**) Relative expression of LINC00982 in 68 pairs of PTC tissues compared with corresponding adjacent normal tissues. (**B**) Relative expression of LINC00982 in PTC patients with different T stage. (**C**) Relative expression of LINC00982 in PTC patients with different TNM stage. (**D**) Relative expression of LINC00982 in PTC patients with or without lymphnode metastasis (lymph node melanomametastasis). (**E**) Relative expression of LINC00982 in PTC patients with or without multifocality. (**F**) Kaplan–Meier OS curves for 68 patients with PTC classified according to relative LINC00982 expression level. ***P<0.001, **P<0.01.

The article "Overexpression of long non-coding RNA LINC00982 suppresses cell proliferation and tumor growth of papillary thyroid carcinoma through PI3K-ATK signaling pathway" was published in 2019. Journal: Biosci Rep.

### Effect of LINC00982 on cell growth *in vitro*

To assess the underlying function and molecular mechanism of LINC00982 in PTC, we first investigated the effect of overexpression or targetted knockdown of LINC00982 on PTC cell proliferation. The expression of LINC00982 in PTC cells was manipulated by LINC00982 overexpression plasmid pcDNA4.0-LINC00982 and terfering plasmids siLINC00982 transfection. Expression of LINC00982 was 16.62-fold and 10.91-fold increase in pcDNA4.0-LINC00982 transfected B-CPAP and BHT101 cells compared with the control vector pcDNA4.0, respectively (Figure 2A), and the endogenous LINC00982 expression was effectively knocked down in siLINC00982 transfected PTC cells compared with siCTRL cells (Figure 2A).

**Figure 2:** Effect of LINC00982 on cell growth *in vitro* (**A**) BHT101 and B-CPAP cells were transfected with pcDNA4.0-LINC00982 and siLINC00982 plasmids, and the expression of LINC00982 was measured by qRT-PCR. (**B**,**C**) CCK-8 assay was conducted to determine the effect of LINC00982 on BHT101 and B-CPAP cell proliferation. (**D**,**E**) EdU stain assay was conducted to determine the effect of LINC00982 on BHT101 and B-CPAP cell proliferation. (**F**,**G**) Colony formation assay was conducted to determine the effect of LINC00982 on BHT101 and B-CPAP cell proliferation. (**H**,**I**) Cell cycle of BHT101 and B-CPAP cells was examined with flow cytometry after pcDNA4.0-LINC00982 and siLINC00982 transfection. ***P<0.001, **P<0.01. *n*=3.

Subsequently, CCK-8, EdU stain, and colony formation assays were conducted to determine the effect of LINC00982 on PTC cell proliferation. As shown in Figure 2B–G, PTC cell proliferation was markedly inhibited by overexpressed LINC00982 and promoted by silenced LINC00982. CCK-8 results showed that the proliferation was significantly inhibited in BHT101 and B-CPAP cells transfected with pcDNA4.0-LINC00982, while markedly promoted in BHT101 and B-CPAP cells transfected with siLINC00982 (Figure 2C,D). Furthermore, the result of EdU assay showed the proliferation of BHT101 and B-CPAP cells was obviously inhibited by pcDNA4.0-LINC00982 and promoted by siLINC00982 (Figure 2E,F). Moreover, colony formation of BHT101 and B-CPAP cells was reduced by pcDNA4.0-LINC00982 and induced by siLINC00982 (Figure 2F,G). Additionally, flow cytometry results showed that overexpression of LINC00982 could increase G1 phase and decrease S phase, and knockdown of LINC00982 could decrease G1 phase and increase S phase in BHT101 and B-CPAP cells (Figure 2H,I). Thus, our results suggested that LINC00982 could control cell cycle to regulate PTC cell proliferation *in vitro*.

The article "Overexpression of long non-coding RNA LINC00982 suppresses cell proliferation and tumor growth of papillary thyroid carcinoma through PI3K-ATK signaling pathway" was published in 2019. Journal: Biosci Rep.

### Effect of LINC00982 on cell migration and invasion *in vitro*

To investigate the effect of LINC00982 on PTC cell migration and invasion, transwell-migration and -invasion assays were performed in BHT101 and B-CPAP cells. Based on the transwell assay results, we found that the migratory and invasive abilities of BHT101 and B-CPAP cells were suppressed by pcDNA4.0-LINC00982, while significantly promoted by siLINC00982 (Figure 3). Therefore, our results indicated that LINC00982 could regulate PTC cell migration and invasion.

**Figure 3:** Effect of LINC00982 on cell migration and invasion *in vitro* The effect of LINC00982 on cell migration and invasion was detected by transwell assay. *** *P<*0.001. *n*=3.

### Overexpression of LINC00982 induces cell apoptosis through PI3K/AKT signaling pathway

According to the above results, LINC00982 could regulate cell proliferation and metastasis *in vitro*. Herein, we further detected the role of LINC00982 on PTC cell apoptosis. Flow cytometry was used to exam cell apoptosis. The apoptosis rate was increased in BHT101 and B-CPAP cells after transfected with pcDNA4.0-LINC00982 and decreased in BHT101 and B-CPAP cells after siLINC00982 transfection (Figure 4A). In addition, western blot results showed that overexpression of LINC00982 could reduce the protein expression of PI3K and phosphorylated AKT (p-AKT), and knockdown of LINC00982 could induce the protein expression of PI3K and phosphorylated AKT (p-AKT) (Figure 4B). Furthermore, the downstream genes of PI3K/AKT signaling pathways, including Bax, Bcl-2, p21, and cyclin D1, were also detected by western blot. As shown in Figure 4B, the protein expression of Bcl-2 and cyclin D1 was reduced, and Bax and p21 was induced in BHT101 and B-CPAP cells after transfected with pcDNA4.0-LINC00982, respectively. While, the protein expression of Bcl-2 and cyclin D1 was induced, and Bax and p21 was reduced in BHT101 and B-CPAP cells after transfected with siLINC00982, separately.

**Figure 4:** Overexpression of LINC00982 induces cell apoptosis through PI3K/AKT signaling pathway (**A**) Apoptosis of BHT101 and B-CPAP cells was examined with flow cytometry after pcDNA4.0-LINC00982 and siLINC00982 transfection. (**B**) Western blot analyzed the protein expression of PI3K, AKT, pAKT, Bax, Bcl-2, p21, and cyclin D1 in BHT101 and B-CPAP cells after pcDNA4.0-LINC00982 and siLINC00982 transfection. ***P<0.001, *P<0.05. *n*=3.

The article "Overexpression of long non-coding RNA LINC00982 suppresses cell proliferation and tumor growth of papillary thyroid carcinoma through PI3K-ATK signaling pathway" was published in 2019. Journal: Biosci Rep.

### LINC00982 inhibits PTC cells tumorigenesis *in vivo*

A xenograft model was established in mice with BHT101 to investigate the antitumor role of LINC00982 *in vivo*. After 4 weeks injection, the tumor volumes were significantly reduced in LINC00982-BHT101 group, while the tumor volumes were markedly induced in siLINC00982-BTH101 group compared with control or NC group (Figure 5A,B). In addition, qRT-PCR results showed that the expression of LINC00982 in LINC00982 formed tumor tissues was significantly higher than control or NC and LINC00982 expression levels in siLINC00982 formed tumor tissues were observably lower than control or NC (Figure 5C). Moreover, western blot results indicated that PI3K, pAKT, p21, and Cyclin D1 had the same expression pattern with the *in vitro* assays (Figure 5D). These results indicate that up-regulation of LINC00982 could inhibit tumor growth and induce apoptosis *in vivo*.

**Figure 5:** LINC00982 inhibits PTC cells tumorigenesis *in vivo* (**A,B**) Xenograft model was constructed to demonstrate the effect of LINC00982 on tumor growth. (**C**) qRT-PCR analyzed the expression of LINC00982 in ectopic tumors. (**D**) Western blot was used to detect the PI3K, AKT, pAKT, Bax, Bcl-2, p21, and cyclin D1 protein expression in ectopic tumors. ***P<0.001. *n*=6.

## Discussion

During the past decades, aberrant expression of lncRNAs has been widely reported in carcinogenesis, and lncRNAs have been regarded as crucial regulators involved in human cancers playing as tumor suppressors or oncogenes. Lan et al. identified that 3499 lncRNAs were differentially expressed in PTC compared with paired non-cancerous tissue, including 1192 up-regulated lncRNAs and 2307 down-regulated lncRNAs using the lncRNA expression microarray [22]. Among the differentially expressed lncRNAs, LINC00982 was considered to be significantly decreased in PCT compared with corresponding pericarcinomatous tissues [23]. Moreover, the antitumor effects of LINC00982 have been established in gastric cancer and lung adenocarcinoma. In the present study, we also observed a decreased expression of LINC00982 in 68 PTC tissues. More important, lower LINC00982 expression was correlated with poorer prognosis in patients with PTC, suggesting the potential antitumous role of LINC00982 in PTC.

An increasing attention focussed on lncRNAs due to their crucial roles in biological processes, including pathogenic processes and normal physiological processes [24–26]. Reportedly, LINC00982 was an independent prognostic factor for gastric cancer patients’ OS and up-regulation of LINC00982 could inhibit gastric cancer growth [13]. Also, Fei et al. found that LINC00982 was decreased in human gastric cancer, and decreased LINC00982 expression was negatively correlated with advanced TNM stage, invasion depth, and regional lymph node metastasis [14]. Overexpression of LINC00982 inhibited renal cancer cell proliferation and induced renal cancer cell apoptosis, and also regulated the PI3K/AKT signaling pathway [16]. LncRNAs have been shown to interact with proteins to influence downstream signaling events. NKILA has been shown to bind to the nuclear factor-κB (NF-κB)/IκB complex, which masks the phosphorylation sites of IκB, thus preventing its degradation [27]. In our present study, we revealed that up-regulation of LINC00982 dramatically inhibited PTC cell proliferation *in vitro*, and the tumor growth *in vivo*, also LINC00982 regulated the PI3K/AKT signaling pathway *in vitro* and *in vivo*, which is consistent with previous studies. Furthermore, whether LINC00980 could bind to the PI3K/AKT pathway need to be further investigated.

The article "Overexpression of long non-coding RNA LINC00982 suppresses cell proliferation and tumor growth of papillary thyroid carcinoma through PI3K-ATK signaling pathway" was published in 2019. Journal: Biosci Rep.

Targetting deregulated signaling pathways in human cancer has been become a potential effective approach in cancer therapy [28]. The phosphatidylinositol 3-kinase (PI3K)/AKT signaling pathway plays a major role in regulating cellular processes, and is also frequently deregulated in human cancers [29]. The PI3K/AKT signaling pathway regulates multiple cellular processes, including cell proliferation [30], apoptosis [31], or cell migration [32]. Tang et al. revealed that lncRNA CRNDE exerts its oncogenic role in hepatocellular carcinoma cell proliferation and growth through regulating PI3K/AKT/GSK3β-Wnt/β-catenin axis [33]. Min et al. demonstrated that up-regulation of LINC00312 decreased thyroid cancer cell proliferation and invasion via suppression of activation of the PI3K/AKT signaling pathway [34]. Overexpression of LINC00982 suppressed renal cancer cell proliferation and induced cell apoptosis via regulating the PI3K/AKT signaling pathway [16]. Here, our study found that overexpression of LINC00982 suppressed cell proliferation and tumor growth *in vitro* and in *vivo*. In addition, our results indicated that LINC00982 played its oncogenic role in PTC cell proliferation and growth by blocking the activation of PI3K/AKT signaling pathway.

In conclusion, our results showed that the expression of LINC00982 was decreased in human PTC tissues and its expression was observably correlated with T stage, TNM stage, lymph node metastasis, and multifocality. Moreover, overexpression of LINC00982 suppressed PTC cell proliferation and induced cell apoptosis *in vitro* and *in vivo*, while, knockdown of LINC00982 promoted PTC cell proliferation and reduced cell apoptosis *in vitro* and *in vivo*. In addition, up-regulation of LINC00982 blocked the activation of PI3K/AKT signaling pathway. All the data indicated that LINC00982 acts as a tumor suppressor gene, and revealed LINC00982-PI3K/AKT signaling pathway regulatory network contributes to PTC. Our results indicated that LINC00982-PI3K/AKT signaling pathway might represent a novel indicator of PTC and might be a potential therapeutic target for diagnosis and therapy.

The article "Overexpression of long non-coding RNA LINC00982 suppresses cell proliferation and tumor growth of papillary thyroid carcinoma through PI3K-ATK signaling pathway" was published in 2019. Journal: Biosci Rep.

## Abbreviations

CCK-8: cell counting kit-8
DMEM: Dulbecco’s modified eagle’s medium
lncRNA: long non-coding RNA
PI3K: phosphatidylinositol 3-kinase
PTC: papillary thyroid cancer
